# Lack of Major Genome Instability in Tumors of p53 Null Rats

**DOI:** 10.1371/journal.pone.0122066

**Published:** 2015-03-26

**Authors:** Roel Hermsen, Pim Toonen, Ewart Kuijk, Sameh A. Youssef, Raoul Kuiper, Sebastiaan van Heesch, Alain de Bruin, Edwin Cuppen, Marieke Simonis

**Affiliations:** 1 Hubrecht Institute, KNAW and University Medical Center Utrecht, Uppsalalaan 8, 3584 CT Utrecht, The Netherlands; 2 Dutch Molecular Pathology Center. Department of Pathobiology, Faculty of Veterinary Medicine, Utrecht University, Yalelaan 1, 3584 CL Utrecht, The Netherlands; Tulane University Health Sciences Center, UNITED STATES

## Abstract

Tumorigenesis is often associated with loss of tumor suppressor genes (such as TP53), genomic instability and telomere lengthening. Previously, we generated and characterized a rat p53 knockout model in which the homozygous rats predominantly develop hemangiosarcomas whereas the heterozygous rats mainly develop osteosarcomas. Using genome-wide analyses, we find that the tumors that arise in the heterozygous and homozygous *Tp53^C273X^* mutant animals are also different in their genomic instability profiles. While p53 was fully inactivated in both heterozygous and homozygous knockout rats, tumors from homozygous animals show very limited aneuploidy and low degrees of somatic copy number variation as compared to the tumors from heterozygous animals. In addition, complex structural rearrangements such as chromothripsis and breakage-fusion-bridge cycles were never found in tumors from homozygous animals, while these were readily detectable in tumors from heterozygous animals. Finally, we measured telomere length and telomere lengthening pathway activity and found that tumors of homozygous animals have longer telomeres but do not show clear telomerase or alternative lengthening of telomeres (ALT) activity differences as compared to the tumors from heterozygous animals. Taken together, our results demonstrate that host p53 status in this rat p53 knockout model has a large effect on both tumor type and genomic instability characteristics, where full loss of functional p53 is not the main driver of large-scale structural variations. Our results also suggest that chromothripsis primarily occurs under p53 heterozygous rather than p53 null conditions.

## Introduction

p53 is regarded as an important gate keeper of genome integrity in healthy cells. In the majority of all tumors the *TP53* gene is mutated and the p53 protein is inactivated [1,2]. Inherited mutations in *TP53* are the cause of Li-Fraumeni syndrome, which is marked by a high incidence of tumors and the development of cancer early in life [3]. Genomic instability can result in different types of large structural rearrangements in the genome. A recent analysis of the Sonic-Hedgehog medulloblastoma brain tumors of Li-Fraumeni patients indicated a strong, permissive connection between *TP53* mutations and chromothripsis, i.e. a massive complex chromosomal rearrangement that occurs in a single event [4]. The exact mechanism of chromothripsis remains elusive but evidence suggests it may occur as a result of chromosome missegregation during cell division and subsequent micronuclei formation [5].

In cancer, cell cycling is often deregulated and accelerated and one of the effects of this rapid cell cycling is telomere shortening. When telomeres become critically short, chromosome end-to-end fusions can occur recurrently, which may result in breakage-fusion-bridges (BFBs) [6]. To maintain telomere length, telomerase or the alternative lengthening of telomeres (ALT) pathway is often activated in tumors and in other cell types that undergo a high rate of cell cycling, like stem cells [7].

Previously, we generated and characterized a rat p53 knockout model in which the homozygous mutant animals completely lack the p53 protein as a result of a C273X nonsense mutation in the sixth exon. This mutation truncates the protein at the DNA binding domain, thereby eliminating functionally essential domains including the nuclear localization domain and the homo-oligomerization domain. The complete absence of functional p53 protein in homozygous mutant animals was demonstrated in embryonic fibroblasts treated with either ultraviolet radiation or doxorubicin [8]. The homozygous rats were found to predominantly develop hemangiosarcomas at about 4 months of age whereas the heterozygous rats mainly develop osteosarcomas at about 8 months of age [8]. This shows that tumor development depends on genotype, but how genotype affects the stability of tumor genomes remains unclear.

In this study we investigate the genomic integrity of the tumor of this p53 mutant rat model, comparing heterozygous and homozygous genotypes. Strikingly, while p53 can be considered the main tumor driver in both genotypes, we find that tumors that are formed in the homozygous p53 knockout animals have a stable tumor genome and are fundamentally different from tumors formed in heterozygous animals, which display extensive chromosomal aberrations and complex structural rearrangements.

## Material and Methods

### Animals

All experiments were approved by the Animal Care Committee of the Royal Dutch Academy of Sciences according to the Dutch legal ethical guidelines. Experiments were designed to minimize the number of required animals and their suffering. The *Tp53* knockout rat (Crl:WI(UL)-Tp53^m1/Hubr^) was generated by target-selected ENU-driven mutagenesis (for detailed description, see [9]). The heterozygous-mutant animal was outcrossed at least 6 times to eliminate confounding effects from background mutations induced by ENU. *Tp53* ^C273X^ rats were bred under standard conditions to generate animals that are heterozygous and homozygous for this allele. Animals were housed under standard conditions in groups of two to three per cage per sex under controlled experimental conditions (12-hour light/dark cycle, 21 ±1°C, 60% relative humidity, food and water ad libitum). Health status and tumor development was monitored weekly. After detection of a visible tumor (age 8–71 weeks) animals were sacrificed.

### Tissue sampling and Rat Embryonic Fibroblasts isolation

The tumor was dissected and split into two: one sample was fixed in 4% neutral buffered formalin for histological analysis and another was snap frozen sample in liquid nitrogen for molecular analysis. DNA extraction was carried out with 20 to 30 mg of snap-frozen and ground tissue using Genomic tips (Qiagen, Venlo, Netherlands). DNA quality was assessed on an agarose gel. If the DNA was degraded, the isolation was repeated. If samples were contaminated with protein or RNA, they were re-isolated using DNeasy spin columns (Qiagen) to ensure high purity of the DNA essential for aCGH and NGS. For rat embryonic fibroblast (REF) isolation heterozygous carriers were mated and at E13.5 embryos were isolated. After washing the embryo thoroughly, the head and visceral organs were removed and used for DNA isolation and genotyping. The embryos were minced and treated with trypsin to get a single cell suspension. REFs were grown in Dulbecco’s modified Eagle’s medium supplemented with 10% fetal calf serum.

### Histological analysis

Immunohistochemistry (IHC) was performed only on those tumors that were undifferentiated on hematoxylin and eosin (HE) stain. The IHC staining procedures were performed according to the protocol of the primary antibody manufacturer. SMA (Abcam (Cambridge, UK) at 1:100), Vimentin (Santa Cruz Biotech (Dallas, TX, USA) at 1:30), Factor VIII (Dako (Santa Clara, CA, USA), 1:500), and Osteocalcin (Merck Millipore (Billerica, MA, USA), 1:400), MyoD-1 (Dako) antibodies were applied overnight in humid chamber at room temperature, then sections were washed and then incubated in (3,3’-diaminobenzidine (DAB) substrate kit for 4 minutes (Vector SK-4100, Vector Laboratories (Burlingame, CA, USA)). Positive and negative control sections were performed for every antibody.

### Western blot

Wild-type and homozygous mutant REFs were treated with 0.5 μM doxorubicin and lysed at 0, 4 and 24 hours after start of treatment and analyzed by Western Blotting using the anti-p53 monoclonal antibody 1C12, which was raised against a synthetic peptide corresponding to residues surrounding Ser20 of human p53 (Cell Signaling Technology, Danvers MA, USA).

### Array Comparative Genomic Hybridization

Array CGH experiments were performed as previously described [10]. Data is available at [NCBI-GEO:GSE55895]. The oligonucleotide design, array fabrication, DNA labeling, hybridization were performed according to manufacturer’s instructions. Microarrays were scanned with a G2565CA scanner (Agilent, Santa Clara, CA, USA) at resolution 2 μm, double pass. Microarray slides were reused once by removing the hybridized probe from the slide (after image acquisition) using the NimbleGen Array Reuse Kit (Roche Nimblegen, Basel, Switzerland). Image analysis was performed using Feature extraction software version 10.5.1.1 (Roche Nimblegen) and CGH-segMNT in NimbleScan 2.6 software (Roche NimbleGen).

#### Gains and losses

Cutoff values for log2 ratio were determined using a control versus control array. Sex and residual chromosomes were excluded from analysis. We defined chromosomal arm-level alteration as a single alteration or an aggregate of alterations that encompass >75% of a chromosomal arm.

#### Chromothripsis

We inferred chromothripsis when we observed at least 10 changes in segmental copy-number involving two or three distinct copy-number states on a single chromosome [4].

#### Breakage-fusion-bridges

We inferred BFB cycles when we observed a stair-like increase in copy-number with multiple segments (minimum of 3 increasing copy-number states) on one side and a single sharp drop on the other side; located at the chromosome start or end.

### Telomere length

500ng of genomic DNA of each tumor was used for SOLiD 5500xl Wildfire (Thermo Fisher Scientific, Life Technologies, Waltham, MA, USA) library preparation and whole genome sequencing resulting in 0.10–1.34x coverage per sample. Reads were mapped onto a telomeric repeat reference (TTAGGG_10_) with BWA 0.5.9 [11] and average telomere length was calculated. Data is available at [NCBI-SRA:PRJEB5836].

### Telomerase and ALT activity

Telomerase activity of tumor cell extracts measured by TRAPeze (TRAPeze XL Telomerase Detection Kit, Merck Millipore). ALT activity of tumor cell extracts was measured by qPCR of CC assay product as previously described [12] and normalized for the ALT-positive control cell line U-2 OS.

## Results and Discussion

We investigated the genetic status of *Tp53* in all tumors found in heterozygous animals by capillary sequencing and found that all tumors show loss of heterozygosity (LOH); data not shown. Thus, all tumors in heterozygous animals have lost the functional *Tp53* allele and have become *Tp53* null.

Next, tumors were histologically examined to determine the tumor-type. In total we excised 26 tumors (10 *Tp53* ^-/-^, 16 *Tp53* ^+/-^) of which 25 could be classified as specific tumor types. In heterozygous animals we found 10 osteosarcomas, 2 fibrosarcomas, 1 leiomyosarcoma, 1 rhabdomyosarcoma and 1 transitional cell carcinoma. In homozygous animals we found 7 hemangiosarcomas, 2 fibrosarcomas and 1 leiomyosarcoma (Table 1). So even though the tumors of all animals do not have functional p53, the tumor spectrum is different between *Tp53* ^*+/-*^ and *Tp53* ^*-/-*^ animals. These results corroborate our previous observation that *Tp53* ^*C273X*^ mutant rats mainly develop sarcomas and that the tumor spectrum of *Tp53* ^*+/-*^ and *Tp53* ^*-/-*^ animals is different. This indicates that the timing of complete p53 loss may affect tumor type. Alternatively, the p53 mutant allele may result in a truncated protein isoform with residual function. Interestingly, a truncated p53 splice isoform was recently described without transcriptional activity but with the ability to attenuate the expression of E-cadherin, similar to certain p53 gain-of-function mutants [13]. The induced premature stopcodon in our rat model results in a truncated protein (30 kDa) that is about 50 amino acids longer than the described p53 isoform (27 kDa). However, western blot analysis did not reveal any indications for the presence of a truncated isoform in doxycyclin treated embryonic fibroblasts of *Tp53* ^*-/-*^ (Fig. 1) [8]. Although the epitope recognized by the antibody used is present in a potential truncated protein, we can not exclude the possibility that a truncated protein is present at undetectable levels. It should be noted, though, that a potential truncated protein due to the C273X mutation would be present in both heterozygous and homozygous mutants and that dominant effects can thus be expected to affect both genotypes.

**Table 1:** Overview of the characteristics of the tumors in mutant *Tp53* rats in this study.

Rat ID	Genotype	Sex	Age (weeks)	Tumor diagnose	Immunohistochemistry	LOH	LOH type	Chromothripsis	Chromothripsis aff. chr.*	BFB cycles	BFB aff. chr.*	Amplified oncogene(s)
196	- / -	Male	21	fibrosarcoma	VM^+^, SMA^–^, OC^–^, F/VIII^–^	-	-	NO	-	NO	-	-
198	- / -	Male	13	fibrosarcoma	VM^+^, SMA^–^, OC^–^, F/VIII^–^	-	-	NO	-	NO	-	-
164	- / -	Male	13	hemangiosarcoma	VM^+^, F/VIII^+^	-	-	NO	-	NO	-	-
174	- / -	Male	18	hemangiosarcoma	ND	-	-	NO	-	NO	-	-
199	- / -	Male	14	hemangiosarcoma	ND	-	-	NO	-	NO	-	-
223	- / -	Female	15	hemangiosarcoma	ND	-	-	NO	-	NO	-	-
261	- / -	Male	12	hemangiosarcoma	ND	-	-	NO	-	NO	-	-
225	- / -	Male	10	hemangiosarcoma	F/VIII^+^	-	-	NO	-	NO	-	-
247	- / -	Male	8	hemangiosarcoma	F/VIII^+^	-	-	NO	-	NO	-	-
201	- / -	Male	20	leiomyosarcoma	VM^+^, SMA^+^, F/VIII^–^	-	-	NO	-	NO	-	-
103	+ / -	Male	54	fibrosarcoma	ND	Yes	deletion	YES	6	NO	-	-
170	+ / -	Male	45	fibrosarcoma	VM^+^, SMA^–^, OC^–^, F/VIII^–^	Yes	deletion	YES	1	YES	7	*Myc*
153	+ / -	Male	49	leiomyosarcoma	VM^+^, SMA^+^, OC^–^, F/VIII^–^	Yes	affected by chromothripsis	YES	10**,13	YES	9	*Vegfa*
20	+ / -	Female	45	osteosarcoma	ND	Yes	gene conversion or copy-neutral SV	NO	-	NO	-	-
82	+ / -	Male	45	osteosarcoma	ND	Yes	gene conversion	YES	7	NO	-	-
97	+ / -	Male	47	osteosarcoma	ND	Yes	affected by chromothripsis	YES	3,8,10**	NO	-	-
100	+ / -	Female	45	osteosarcoma	ND	Yes	gene conversion or copy-neutral SV	NO	-	NO	-	-
112	+ / -	Female	71	osteosarcoma	ND	Yes	affected by chromothripsis	YES	3,10**	YES	6, 10	*Mycn*, *Alk*
118	+ / -	Male	41	osteosarcoma	ND	Yes	gene conversion	NO	-	NO	-	-
142	+ / -	Male	54	osteosarcoma	ND	Yes	deletion	YES	5	YES	9	*Vegfa*
144	+ / -	Male	68	osteosarcoma	ND	Yes	deletion	NO	-	YES	5, 7	*Myc*
160	+ / -	Female	52	osteosarcoma	ND	Yes	deletion	NO	-	NO	-	-
202	+ / -	Male	34	osteosarcoma	ND	Yes	deletion	YES	10,17	YES	14	-
9	+ / -	Female	36	rhabdomyosarcoma	MYD^+^, F/VIII^+^	Yes	gene conversion or copy-neutral SV	YES	6	NO	-	-
125	+ / -	Female	46	transitional cell carcinoma	ND	Yes	gene conversion or copy-neutral SV	NO	-	NO	-	-
95	+ / -	Male	54	ND	ND	Yes	deletion	NO	-	NO	-	-

* Affected chromosomes

** *Tp53* locus affected

ND: not determined, LOH: loss of heterozygosity, SV: structural variant, VM: Vimentin, OC: Osteocalcin, SMA: smooth muscle actin, F/VIII: factor VIII, MYD: MyoD-1.

^+^: Positive IHC staining,

^–^: negative IHC staining

**Fig 1:** *Tp53* ^*C273X*^ results in a complete lack of p53 protein. (**a**) Schematic representation of the normal and truncated rat p53 protein and the p53 isoform as described in [13]. The epitope of the antibody used in (b) is indicated with an asterisk. (**b**) Western blot analysis of wild type and *Tp53* ^*C273X*^ mutant Rat Embryonic Fibroblasts (REFs) treated for 0,4 and 24 hours with doxorubicin and analyzed using Western Blotting.

To investigate whether absence of p53 affects genomic stability in the tumors, we performed array comparative genomic hybridization (aCGH) on tumor versus control tissue to detect copy number variants (CNVs) (S1 Fig.). First, we investigated the presence of aneuploidies in the tumors. We defined an aneuploidy as an event in which at least 75% of a chromosome or chromosomal arm was affected and the copy-number status throughout the affected region was the same. We found a clear difference in the number of aneuploidy events between tumors that arise in heterozygous rats compared to those in homozygous rats: contrary to our expectations, tumors from homozygous animals show almost no deleted or gained chromosomes whereas tumors from heterozygous animals display massive aneuploidies (Fig. 2a). Next, we counted all base pairs that are affected by CNVs (excluding the aneuploidies) in tumors from homozygous animals to tumors of heterozygous animals. Strikingly, we find that in homozygous tumors, in addition to the absence of chromosomal events, also less base pairs are affected by CNVs (Fig. 2b). In heterozygous rats, we observed highly aneuploid and CNV-rich genomes in osteosarcomas, in line with known human osteosarcoma genomic profiles [14]. Although the main tumor type observed in homozygous animals, hemangiosarcomas, is also reported to harbor many aneuploidies in human [15], we identified only three gained or lost chromosomes in seven hemangiosarcomas. A typical example of the type and amount of aberrations observed in osteosarcomas and hemangiosarcomas is shown in Fig. 2c. These data indicate that in this rat p53 knockout model, genomic instability is not a prerequisite for tumor formation when p53 is already completely inactivated, but also that complete absence of p53 does not systematically induce large-scale genomic instability.

**Fig 2:** Tumors from homozygous *Tp53* ^*C273X*^ mutant rats show significantly less CNVs than tumors from heterozygous *Tp53* ^*C273X*^ rats. (**a**) Counts of fully gained or lost chromosomes (>75%) from array CGH data on tumors DNA versus healthy control DNA. Tumors from heterozygous animals (n = 16) and tumors from homozygous animals (n = 10) were compared using a Student’s *t*-test. (**b**) A sum of all altered base pairs (gained or lost) per tumor. Tumors from heterozygous animals (n = 16) and tumors from homozygous animals (n = 10) were compared using a Student’s *t*-test. (**c**) Two representative examples of the aCGH data. The upper panel shows the amount of CNVs in the genome of an osteosarcoma from a heterozygous animal (Rat ID 112); the lower panel shows CNVs in a hemangiosarcoma from a homozygous animal (Rat ID 261).

Recently, a link between *TP53* mutation status and the presence of chromothripsis has been postulated [4]. Therefore we set out to explore the presence of chromothripsis events in the tumors under study. In chromothripsis, one or a few genomic regions in the genome are randomly shattered and reassembled. To infer the occurrence of chromothripsis, we used the definition put forward by Rausch et al [4], which requires at least ten changes in segmental copy-number involving two or three distinct copy-number states on a single chromosome. In nine out of sixteen tumors from heterozygous rats we find evidence of chromothripsis (Fig. 3a and Fig. 3b). In contrast, none of the tumors from homozygous rats display any evidence for chromothripsis. Our results support the previous finding that heterozygous p53 mutations increase the incidence of chromothripsis. Question remains what the order of events is; is loss of the functional *Tp53* allele necessary to elicit genomic instability, which then results in chromothripsis? The finding that none of the homozygous tumors display chromothripsis suggests that complete loss of p53 is not the main driver to elicit this type of genomic rearrangement. From our data, it appears more likely that the loss of one allele of p53 makes cells more sensitive to (some forms) of genomic instability. Resulting rearrangements subsequently result in loss of the healthy p53 allele and further tumor development. In support of this view we find in the aCGH data that in three out of nine chromothripsis cases the second *Tp53* allele is lost via this mechanism (Table 1).

**Fig 3:** Tumors from homozygous *Tp53* ^*C273X*^ mutant rats do not show any evidence for the occurrence of chromothripsis. (**a**) Chromothripsis signatures were counted in aCGH data from tumors from heterozygous animals (n = 16) and tumors from homozygous animals (n = 10). (**b**) Representative examples of chromothripsis in three different tumors from heterozygous animals. The lower panel shows LOH of the *Tp53* locus as a result of chromothripsis.

Chromothripsis is potentially linked to the occurrence of another hallmark of cancer and genomic instability: breakage-fusion-bridges (BFB) cycles, including gene amplifications [16]. As a consequence of BFB cycles a distinct stair-like gradient of copy-number increasing genomic segments are formed which can be detected by array CGH[17]. We therefore explored our data for such signatures and identified BFB cycle events in six out of sixteen tumors, all formed in heterozygous rats (Fig. 4a). All chromosomes with a BFB cycle-signature contained highly amplified segments with well-known oncogenes like *Myc*, *Mycn*, *Vegfa* and *Alk* (Fig. 4b and Table 1). In tumors from homozygous animals however, we did not find any evidence for BFB cycles. BFB cycles are caused by telomeric shortening and subsequent crisis and might play a role in the occurrence of chromothripsis [16]. However, while five out of six BFB events were found in tumors that also contained chromothripsis events, there is not a full correlation between these events and the chromosomes affected by both events overlap only in a single case. This argues against a direct mechanistic link between BFB and chromothripsis event, although indirect effects or a common driver can not be excluded.

**Fig 4:** Tumors from homozygous *Tp53* ^*C273X*^ mutant rats never show evidence for the occurrence of BFB cycles. (**a**) BFB cycle signatures were counted in aCGH data from tumors from heterozygous animals (n = 16) and tumors from homozygous animals (n = 10). (**b**) Representative examples of BFB cycles in two different tumors from heterozygous animals. Both panels show a gene amplification of the *Myc* oncogene on chromosome 7.

Most examples of chromothripsis observed by Stephens et al [16] involve regions extending to the telomeres. Next to this, chromothripsis is found mainly in older patients [18]. We thus hypothesized that the relative stability of p53 null tumors depends on activated telomere-lengthening mechanisms that protect against BFBs and potentially chromothripsis in the tumors of homozygous animals. Therefore, we interrogated telomere length of the tumor cells by next-generation sequencing. We counted and normalized the reads that mapped to the telomeric repeat (TTAGGG) and calculated the length of an average telomere per sample. Tumors of homozygous animals showed significantly longer telomeres compared with tumors of heterozygous animals (p<0.05) or with ear control DNA (p<0.01, Student’s t-test) (Fig. 5a). This suggests that telomere length may indeed be a factor that is involved in the difference in genomic rearrangements. Of note, the telomeric length of rat (20–100 kb [19]) differs from mouse (40–60kb [20]) and human (10 kb [20]). So cautiousness should be applied when comparing these organisms. However, the differences between the two heterozygous and homozygous *Tp53* genotypes in this study is noteworthy. This difference can be caused by increased shortening in the heterozygous tumors, or activated telomere lengthening in the homozygous background tumors. We measured the presence of the two main telomere lengthening pathways in the tumors by quantifying telomerase activity and the amount of C-circles, which are a measure for the activity of the alternative lengthening of telomeres (ALT) pathway [21]. We found that in only one out of nine homozygous tumors a telomere lengthening pathway was clearly activated (Fig. 5b and Fig. 5c). Thus, activation of known mechanisms of telomere lengthening are not a likely cause of the stable genomes in the homozygous animals. It is possible that these tumors have an alternative method to maintain telomere length, or that the difference in telomere length reflects telomeric shortening in the heterozygous animals.

**Fig 5:** Tumors from homozygous *Tp53* ^*C273X*^ mutant rats show significantly longer telomeres than tumors from heterozygous *Tp53* ^*C273X*^ rats. (**a**) Length of an average telomere per tumor. Tumors from heterozygous animals (n = 16) and tumors from homozygous animals (n = 10) were compared using a Student’s *t*-test. (**b**) Telomerase activity of tumor cell extracts, normalized for the telomerase-positive control cell line provided with the kit. Error bars represent s.e.m. (**c**) ALT activity of tumor cell extracts, normalized for the ALT-positive control cell line U-2 OS.

In summary, we show that the tumors in p53 heterozygous and homozygous mutant rats are different in many aspects. As described before [8] the tumor spectrum is different. Homozygous animals mainly develop hemangiosarcomas between 2 and 5 months of age, whereas heterozygous animals mainly develop osteosarcomas between 8 and 16 months of age. Our data show that this early occurrence of these tumors is not due to increased genomic instability. On the contrary, tumors from homozygous animals contain a low number of aneuploidies and CNV affected base pairs. Furthermore these tumors do not display any complex structural aberrations such as chromothripsis and BFB cycles. Although the observed differences between the genotypes is evident, we have to keep in mind that the different tumor types per genotype may play a role in this observation. The genomes were particularly stable in the hemangiosarcomas. In this respect, it is relevant to look at the cell type of origin of hemangiosarcomas: the hemangioblasts [22–24]. Hemangioblasts are progeny from the bone-marrow-derived hematopoietic stem cells (HSCs). Stem cells, like HSCs, are known to actively maintain their telomeres, since they continuously produce progeny and thus cycle throughout life. In p53 null mice, HSCs expand and proliferate greatly and their apoptotic potential is reduced [25,26]. The high proliferation rate in p53 null animals in combination with the telomere maintenance potential may explain the observed hemangiosarcoma tumors with a stable genome.

## Conclusions

Overall our results underscore the principle of common sequence of oncogenic events in tumorigenesis [27]. These data show that the mere loss of functional p53 is not sufficient to induce large-scale genomic instability in this rat p53 knockout model.

## Supporting Information

S1 Fig Overview of all aCGH experiments in this study. On the x-axis, each color represents a separate chromosome. Log2 ratios are plotted on the y-axis.
(TIF)
